This article has been retracted.

# Detection of CEA and ProGRP Levels in BALF of Patients with Peripheral Lung Cancer and Their Relationship with CT Signs

**DOI:** 10.1155/2022/4119912

**Published:** 2022-07-27

**Authors:** Kui Tian, Zhengmin Li, Lixin Qin

**Affiliations:** Department of Radiology, Wuhan Pulmonary Hospital, Wuhan, 430000 Hubei Province, China

## Abstract

**Background:**

Lung cancer is a common clinical thoracic malignant tumor, which had a serious impact on the safety of patients, currently ranking first in all malignant tumors in morbidity and mortality, with generally less than 5% survival rate in 5 years.

**Objective:**

To investigate the relationship and significance between carcinoembryonic antigen (CEA) and precursor gastrin-releasing peptide (ProGRP) changing levels in bronchoalveolar lavage fluid (BALF) and CT imaging features in patients with peripheral lung cancer.

**Methods:**

A total of 90 patients diagnosed with peripheral lung cancer as the lung cancer group and 60 patients with benign lung diseases as the control group in our hospital from May 2019 to October 2021 were selected to compare the differences of CEA and ProGRP in BALF by the classification of CT features.

**Results:**

The levels of CEA and ProGRP in the BALF of the lung cancer group were significantly higher than those of the control group; the proportion of patients with lobulation sign, burr sign, ground glass sign, pleural effusion, and lesion diameter ≥ 3.0 cm in the lung cancer group was higher than that in the control group; the CEA level in BALF of lung cancer patients with spicule sign, pleural effusion, and lesion diameter ≥ 3.0 cm was significantly higher than that without these symptoms, while ProGRP level in the BALF of lung cancer patients with lobulation sign, burr sign, ground glass sign, pleural effusion, and lesion diameter ≥ 3.0 cm was significantly higher than that of lung cancer patients without these symptoms.

**Conclusion:**

The check of CEA and ProGRP in BALF in combination with CT features has a certain clinical value for the diagnosis of lung cancer. At the same time, the increased levels of CEA and ProGRP in BALF have a certain correlation with the changes of malignant signs of lung cancer in CT examination.

## 1. Introduction

As a common malignant tumor, lung cancer is easy to be missed and misdiagnosed due to the atypical early clinical signs of patients; thus, early diagnosis and treatment of lung cancer are of great significance for improving the prognosis of patients. At present, there are many methods for clinical diagnosis of lung cancer, with CT examination as a more common way in clinical practice. However, the diagnosis rate is not high in some patients with peripheral and adjacent pleura [1]. In recent years, bronchoscopy has played an important role in the diagnosis of lung cancer. The monitoring of tumor-related markers by bronchoalveolar lavage after aspiration of local bronchoalveolar fluid can avoid the disadvantage of low sensitivity of serological indicators. The content of related markers in alveolar fluid usually appears earlier, and the concentration is high. CEA is a commonly used clinical serological tumor marker which will significantly increase in patients with various malignant tumors. The expression of ProGRP and the precursor of gastrin-releasing peptide with high stability, have been confirmed to be elevated in lung cancer patients, while malignant tumors can produce ProGRP to promote tumor reproduction and metastasis in an autocrine manner [2]. At present, there is no clinical report on the relationship between the levels of CEA and ProGRP in BALF and CT imaging features in patients with lung cancer. In order to further improve the diagnosis accuracy of lung cancer and accurately evaluate the prognosis of patients, this study has analyzed about it, and the report is as follows.

### 1.1. Core Tips

Even the early surgical treatment can prolong the survival of patients, as one of the malignant tumors with high clinical incidence, lung cancer has already developed in the advanced stage when seeing the doctor due to the atypical early clinical signs of some patients. Pathological examination is the gold standard for diagnosing lung cancer, but the trauma is relatively large with a poor specificity of CT and other imaging tests. With the development of bronchoscopy, which obtains bronchoalveolar lavage fluid and takes molecular biological diagnosis into clinical practice, analyzing the concentration of specific tumor markers in patients' bronchoalveolar lavage fluid has certain value for the early diagnosis of lung cancer. However, it is rarely used in patients in this region. This study relied on this to analyze by using bronchoalveolar lavage fluid tumor-related markers and screened specific indicators for the diagnosis of lung cancer, thus improving the clinical efficacy for early diagnosis of it.

## 2. Materials and Methods

### 2.1. General Information

A total of 90 patients diagnosed with peripheral lung cancer as the lung cancer group and 60 patients with benign lung diseases as the control group in Wuhan Pulmonary Hospital from May 2019 to October 2021 were selected.

Inclusion criteria were as follows: (1) patients from 19 to 75 years old; (2) the diagnosis of peripheral lung cancer patients was confirmed by pathological examination after lung puncture or bronchoscopy or postoperative pathological examination in line with the standard in “Clinical Oncology Society (CSCO) Guidelines for the Diagnosis and Treatment of Primary Lung Cancer” [3]; (3) patients with benign lung tumors were pathologically confirmed as inflammatory nodules, fibroids, etc.; (4) all patients have underwent pulmonary lavage examination and chest CT examination; and (5) the research program meets the requirements of the medical ethics expert group of our hospital. The research program is approved by patients and their families, and they signed informed consent.

Exclusion criteria were as follows: (1) history of radiotherapy, chemotherapy, and immunological therapy for lung tumors; (2) recurrent lung tumors after previous surgery; (3) lactating women; (4) metastasis to the lungs due to other malignant tumors; and (5) accompanied by major diseases of other systems.

### 2.2. Bronchoalveolar Lavage and Index Detection Methods

When the intravenous compound anesthesia was satisfied, with the supine position, an Olympus BF-F260 electronic bronchoscope was inserted into the patient's nose. The distal end of the bronchoscope was placed near the bronchial opening above the lesion, and 1-2 mL of 2% lidocaine was injected through the biopsy hole to lavage the lung segment. Then, 60-120 mL of normal saline at 37°C was injected through the operation channel, using a controllable suction tube to obtain bronchoalveolar fluid. After filtering out the mucus and storing it in a 4°C refrigerator, 10 mL of the liquid was centrifuged at 1200 r/min for 10 min, and the concentration of CEA and ProGRP was determined by enzyme-linked immunosorbent assay, with Hitachi providing 7600i automatic biochemical analyzer for determination and Beijing Northern Institute of Biotechnology providing detection kits.

### 2.3. CT Scan Examination

The instrument used was as follows: LightSpeed VCT64 row CT provided by GE Company in the United States to carry out inspection and parameter settings: tube voltage 120 kv, tube current 300 mAs, layer thickness 5 mm, layer spacing 5 mm, scanning time 5-7 s, and matrix 512 × 512. In combination with the images, two physicians with more than 5-year experience in imaging conducted a double-blind analysis to evaluate the location, size, shape, number, and extent of the lesions and the final diagnosis was made after consultation if they held different opinions.

### 2.4. Statistical Processing

The measured values of CEA and ProGRP in the BALF of the patients in this study were tested by normal distribution, and they were all in line with the approximate normal distribution or normal distribution, expressed as ($\bar{x}\pm s$), and the *t* test was used for comparison between the two groups; the *χ*^2^ test was used to compare the nonranked count data between groups; professional SPSS21.0 software was used for data processing, and the test level was *α* = 0.05.

## 3. Results

### 3.1. Comparison of Baseline Data between the Two Groups of Patients

The age, BMI, gender, smoking, drinking, and comorbidities of the lung cancer group and the control group were compared to show that there was no significant difference in the above data between the two groups, which was balanced and comparable and met the requirements of clinical research data (*P* > 0.05) (Table 1).

### 3.2. Comparison of CEA and ProGRP Levels in BALF between Two Groups

The levels of CEA and ProGRP in the BALF of the lung cancer group were significantly higher than those of the control group with statistical significance (*P* < 0.05) (Table 2, Figure 1).

### 3.3. Comparison of CT Imaging Features between the Two Groups

The proportion of patients with lobulation sign, burr sign, ground glass sign, pleural effusion, and lesion diameter ≥ 3.0 cm in the lung cancer group was higher than that in the control group (Table 3).

### 3.4. Comparison of CEA and ProGRP Levels in BALF of Lung Cancer Patients with Different CT Imaging Features

The CEA level in BALF of lung cancer patients with spicule sign, pleural effusion, and lesion diameter ≥ 3.0 cm was significantly higher than that without these symptoms, with statistically significant difference (*P* < 0.05), while ProGRP level in the BALF of lung cancer patients with lobulation sign, burr sign, ground glass sign, pleural effusion, and lesion diameter ≥ 3.0 cm was significantly higher than that of lung cancer patients without these symptoms, with statistically significant difference (*P* < 0.05) (Table 4).

## 4. Discussion

Lung cancer is mainly caused by abnormal proliferation of malignant tumor cells. The main clinical signs are abnormal tumors in the lung. Due to the imbalance of cell growth regulation in vivo and abnormal proliferation of malignant tumor cells, local infiltration and distant metastasis are two important characteristics [3]. With the development of modern diagnostic methods, the bronchoalveolar lavage method can improve the clinical diagnostic efficiency by collecting the alveolar surface fluid and diagnosing the relevant markers. The relevant markers in the bronchoalveolar lavage fluid appear earlier and have high concentrations, thus becoming an emerging clinical diagnostic method [4, 5]. In this study, the levels of CEA and ProGRP in the BALF of the patients with lung cancer were significantly higher than those of the control group, indicating that the levels of CEA and ProGRP were significantly increased in patients with lung cancer.

As a soluble glycoprotein, CEA is the most common in the fetal gastrointestinal tract. It is known to exist in embryonic tissues and malignant tumor cells and generally reduce after the fetus is born. CEA is more sensitive to adenocarcinoma; as a result, it has important value in the diagnosis of various malignant tumors [6].

The increase in the concentration of CEA in BALF is generally due to the accumulation of CEA produced by the metabolic secretion of tumor cells in the lesion site, and the release into the blood and body fluids leads to a significant increase in the content. However, the liver can degrade CEA in our blood; thus, CEA concentrations in part of the lung were significantly higher than those in blood [7, 8].. Some scholars have found that the CEA concentration of malignant lesions in lung cancer patients' BALF is significantly increased. Besides, the positive rate of patients at stages I and II is significantly lower than that of patients at stages III and IV, confirming that the concentration of CEA in bronchoalveolar lavage fluid is higher and appears earlier. It is considered that the products formed by the metabolism of tumor cells are restricted and secreted to the cell surface, then enter the bronchi, and finally enter the blood. Therefore, the early detection of CEA in serum is low, resulting in a large difference in serum and alveolar content, which is basically the same as the results of this study [9].

Some scholars have reported that tumor cells in patients with small cell lung cancer can synthesize and release GRP, which mainly proliferate tumor cells by autocrine or cell-to-cell interaction. Therefore, the detection of GRP can reflect the occurrence and development of small cell lung cancer, but GRP is unstable in serum with a half-life of only 2 min, so it is difficult to be detected, while ProGRP is relatively stable, and its monitoring can represent GRP levels and GRP gene expression [10]. Some clinical scholars have reported that serum ProGRP is a relatively specific tumor marker for small cell lung cancer. It may be related to the tendency of endocrine differentiation in some NSCLC; thus, it has an ordinary sensitivity and specificity. ProGRP was significantly elevated in BALF, which has a certain value for clinical diagnosis of lung cancer [11].

CT has always been an important method for clinical diagnosis of lung cancer. In this study, the proportion of patients with lobulation sign, spiculation sign, ground glass sign, pleural effusion, and lesion diameter ≥ 3.0 cm in the lung cancer group was higher than that in the control group. The lobulation sign is the most common one in lung cancer, which generally has an arc-shaped convexity tumor. The concave interphase of the arc results in the lobulated masses, which is mainly due to the uneven growth rate of each part of the tumor edge and different resistance in the growth process, especially the deep lobulation sign that is of great value in the diagnosis of lung cancer; the burr sign, the appearance of radial short, thin, and rigid shadows around the lung tumor, is on the one hand due to the infiltration of tumor cells into the bronchi and blood vessels, and on the other hand, the proliferation of fibrous tissue of malignant tumors will cause scar contraction burr sign [12]; the ground glass sign is the formation of a glass density shadow around the tumor. In peripheral lung cancer, it indicates the infiltration of tumor cells into the interstitium, but it can also appear in some hemorrhagic and infectious lesions, so the specificity of the diagnosis of lung cancer is relatively low; lesions with a diameter of ≥3.0 cm are easier to diagnose clinically, mainly because the larger the tumor volume, the greater the impact on the CT value due to the change in blood vessel density. The high degree of tumor invasion and the abundance of blood vessels resulted in the significant increase of CT value [13]. Lung cancer generally shows invasive growth, with short and thin burrs facing the surrounding depths, so the formation of a hyperplasia reaction leads to the contraction of the pleura, and finally, a dead space containing liquid is formed between the visceral and parietal pleura. At the same time, due to the necrosis of tumor cells, the fluid depth is more likely to form pleural effusion [14].

In this study, the relationship between CT features and the concentrations of CEA and ProGRP in BALF was analyzed to find that the levels of CEA and ProGRP in BALF of lung cancer patients with burr sign, pleural effusion, and lesion diameter ≥ 3.0 cm were significantly increased, showing that there was a certain relationship between CT features and CEA and ProGRP levels in patients with lung cancer. The lesions of lung cancer are irregular and the edge is not clear, which can distinguish benign and malignant tumors. The edge of the lesion is short burr, accompanied by pleural effusion, and other conditions will cause the edge of the lesion to be unclear. It is suggested that lung cancer growth is invasive and can invade adjacent tissues and blood vessels; thus, the detection of related tumor markers in BALF will increase more significantly, which is consistent with the results of this study [15]. The increasing tumor diameter suggested that tumor cells had stronger proliferative ability, poorer prognosis, and higher concentration of tumor markers in vivo. Tumor cells in patients with spiculation and pleural effusion will form relatively independent tumor cell subsets, suggesting that they have high malignant biological behavior [16–20].

This study analyzed the CT imaging features of peripheral lung cancer patients and observed the concentrations of CEA and ProGRP in BALF to learn the imaging specificity of peripheral lung cancer and the tumor markers in BALF, which laid a certain foundation for early diagnosis of lung cancer. At the same time, the relationship between imaging features and molecular biological markers was preliminarily discussed to associate imaging examination with tumor molecular biological examination methods. It has certain value to explain the diversity and complexity of tumors, and is helpful to guide the clinical selection of reasonable treatment plans. However, due to the small number of cases included in this study, it is not possible to further analyze the imaging characteristics and molecular biological indicators of patients with different tumor stages and clinicopathological types. Meanwhile, it is not possible to discuss the influencing factors of different tumor stages and pathological types; thus, it is necessary to increase the sample size and the observation index to further demonstrate in the future.

In summary, the check of CEA and ProGRP in BALF in combination with CT features has a certain clinical value for the diagnosis of lung cancer. At the same time, the increased levels of CEA and ProGRP in BALF have a certain correlation with the changes of malignant signs of lung cancer in CT examination.

## Figures and Tables

**Figure 1:** Histogram of CEA and ProGRP levels in BALF between two groups.

**Table 1:** Comparison of baseline data of two groups of patients.

Group	*n*	Age (years)	BMI (kg/m^2^)	Gender (%)		Smoking (%)	Drinking (%)	Concomitant disease		
				Male	Female			Hypertension	Diabetes	Hyperlipidemia
Lung cancer group	90	66.21 ± 6.83	23.63 ± 1.86	56 (62.22)	34 (37.78)	29 (32.22)	31 (34.44)	26 (28.89)	12 (13.33)	34 (37.78)
Control group	60	67.84 ± 7.40	23.48 ± 1.70	31 (51.67)	29 (48.33)	16 (26.67)	12 (20)	12 (20)	4 (6.67)	21 (35)
*t*/*χ*^2^		-1.385	0.501	1.647		0.529	3.673	1.504	1.679	0.120
*P*		0.168	0.617	0.199		0.467	0.055	0.220	0.105	0.729

**Table 2:** Comparison of CEA and ProGRP levels in BALF between two groups.

Group	*n*	CEA (*μ*g/L)	ProGRP (pg/mL)
Lung cancer group	90	63.84 ± 13.20	148.32 ± 18.46
Control group	60	7.84 ± 2.01	22.03 ± 4.38
*t*		32.575	51.972
*P*		0.000	0.000

**Table 3:** Comparison of CT imaging features between two groups (*n* (%)).

CT imaging features	Lung cancer group (*n* = 90)	Control group (*n* = 60)	*χ* ^2^	*P*
Lobulation sign (%)			10.679	0.001
Yes	56 (62.22)	21 (35.00)		
No	34 (37.78)	39 (65.00)		
Burr sign (%)			10.670	0.001
Yes	34 (37.78)	8 (13.33)		
No	56 (62.22)	52 (86.67)		
Vacuolation sign (%)			2.778	0.096
Yes	14 (15.56)	16 (26.67)		
No	76 (84.44)	44 (73.33)		
Ground glass sign (%)			7.462	0.006
Yes	39 (43.33)	13 (21.67)		
No	51 (56.67)	47 (78.33)		
Pleural effusion (%)			10.070	0.002
Yes	27 (30.00)	5 (8.33)		
No	63 (70.00)	55 (91.67)		
Lesion diameter (%)			12.430	0.000
≥3.0 cm	32 (35.56)	6 (10.00)		
<3.0 cm	58 (64.44)	54 (90.00)		

**Table 4:** Comparison of CEA and ProGRP levels in BALF of lung cancer patients with different CT imaging features ($\bar{x}\pm s$).

CT imaging features	*n*	CEA (*μ*g/L)	*t*	*P*	ProGRP (pg/mL)	*t*	*P*
Lobulation sign (%)			0.889	0.376		2.494	0.014
Yes	56	64.78 ± 12.87			151.70 ± 16.90		
No	34	62.29 ± 12.90			142.75 ± 15.82		
Burr sign (%)			2.109	0.038		3.612	0.001
Yes	34	67.43 ± 11.65			156.65 ± 15.14		
No	56	61.66 ± 13.11			143.26 ± 18.10		
Vacuolation sign (%)			-0.758	0.450		-0.694	0.489
Yes	14	61.50 ± 10.03			145.25 ± 12.83		
No	76	64.27 ± 12.95			148.89 ± 18.78		
Ground glass sign (%)			0.765	0.447		4.623	0.000
Yes	39	65.02 ± 12.76			157.76 ± 16.28		
No	51	62.94 ± 12.81			141.10 ± 17.43		
Pleural effusion (%)			2.614	0.011		2.900	0.005
Yes	27	68.94 ± 10.43			156.20 ± 14.94		
No	63	61.65 ± 12.77			144.94 ± 17.63		
Lesion diameter (%)			3.935	0.000		5.288	0.000
≥3.0 cm	32	71.08 ± 13.14			161.44 ± 15.00		
<3.0 cm	58	59.85 ± 12.86			141.08 ± 18.70		

## Data Availability

The datasets used and analyzed during the current study are available from the corresponding author upon reasonable request.
